The article "Proteochemometric Method for pIC50 Prediction of Flaviviridae" was published in 2022. Journal: Biomed Res Int.

# Proteochemometric Method for pIC50 Prediction of Flaviviridae

**DOI:** 10.1155/2022/7901791

**Published:** 2022-09-15

**Authors:** Divye Singh, Avani Mahadik, Shraddha Surana, Pooja Arora

**Affiliations:** Engineering for Research, Thoughtworks Technologies, Pune, Maharashtra 411006, India

## Abstract

Viruses remain an area of concern despite constant development of antiviral drugs and therapies. One of the contributors is the Flaviviridae family of viruses causing diseases that need attention. Among other anitviral methods, antiviral peptides are being studied as viable candidates. Although antiviral peptides (AVPs) are emerging as potential therapeutics, it is important to assess the efficacy of a given peptide in terms of its bioactivity. Experimental identification of the bioactivity of each potential peptide is an expensive and time consuming task. Computational methods like proteochemometric modeling (PCM) is a promising method for prediction of bioactivity (pIC50) based on peptide and target sequence pair. In this study, we propose a prediction of pIC50 of AVP against the Flaviviridae family that may help make the decision to choose a peptide with desired efficacy. The peptides data was collected from a public database and target sequences were manually curated from literature. Features are calculated using peptide and target sequence PCM descriptors which consist of individual and cross-term features of peptide and respective target. The resultant *R*^2^ and MAPE values are 0.85 and 8.44%, respectively, for prediction of pIC50 value of AVPs.

## 1. Introduction

Viral diseases have been a cause of multiple epidemic outbreaks in the last few decades. This includes many different viruses like Ebola, Zika, Dengue, SARS, and others. Although belonging to one bigger group of viruses, they differ a lot in their activity, sequence, structure, and function. Viruses are also known to have continuous mutations, which makes it necessary and complex to identify antiviral drug candidates. This leads to the need for continuous drug development. Recently, peptide-based antivirals have gained a lot of importance and have shown promising development [1]. In this work, we study methods to predict the pIC50 value for the Flaviviridae family. Among various types of viruses, publically available data is found majorly for hepatitis C virus (HCV) and dengue virus (DENV). Rajput and Kumar developed an algorithm to identify inhibitory activity of chemicals from ChEMBL and peptides from AVPpred databases against Flaviviruses using QSAR method [2]. Recently, Geoffrey et al. developed machine learning based Auto-QSAR using PubChem data, which generated drug leads for Flaviviruses. For the drug leads and their target proteins in silico modeling was performed [3].

The article "Proteochemometric Method for pIC50 Prediction of Flaviviridae" was published in 2022. Journal: Biomed Res Int.

Generally, antiviral peptides are studied based on physicochemical properties, evolutionary properties, and profiles based on only peptide attributes [4]. However, a peptide can have good physicochemical properties that are similar to other bioactive peptides but its efficacy cannot be identified unless its bioactivity is experimentally determined. The inhibition constant (IC) 50 value is commonly used for validating the activity of a peptide. Experimental determination of IC50 is an expensive and tedious task. Taking all the potential peptides for experimental validation might not be feasible. Prediction of IC50 values can reduce the time and effort and help in selecting the most promising peptide for further experimentation. There is very little research done in the area of in silico methods for IC50 value prediction. To understand the IC50 of a peptide, it is necessary to understand the interaction with the target protein. One method for doing so is proteochemometric modelling (PCM).

PCM is a computational method that can predict the bioactivity relations between ligand and targets. It is a method to incorporate the target interaction into sequence-based analysis. Three types of descriptors are included in PCM-Target descriptor (captures information of target), Ligand descriptor (captures information of ligand), and Cross-term descriptor (captures interaction between the ligand and its target). With the different types of interactions studied, the scope of PCM has expanded to include protein-peptide, protein-DNA, and protein-protein interactions.

### 1.1. Literature Survey

Recently, Parks et al. using the ChEMBL25 dataset, generated proteochemometric models to predict pIC50 using random forest and feed-forward neural network [5]. The study checked the usability of PCM model to classify binders and nonbinders. For the ChEMBL25 data set, various physicochemical properties like log P, molecular weight, number of specific bonds, and fingerprints were used as descriptors. Yordanov et al. demonstrated the use of PCM for analysing the structure-affinity relationship of antigen peptides binding to HLA-DP proteins [6]. The HLA system plays an important part in the immune system. The HLA proteins bind to a wide range of antigenic peptides, which is essential for the immune recognition of the antigens. The chemical structures of peptides and proteins used were described by three z-scales. Bio-activity modeling of multiple compounds against protein isoforms was done by Rasti et al. using proteochemometrics modeling [7]. They applied PCM to investigate inhibition of Carbon Anhydrase isoforms using a combination of different descriptors (three z-scale, five z-scale and, GRIND). Mutations affect the antimicrobial activity. The PCM model has also been used to identify the mutations. The study by Nabu et al. helped in understanding the impact of physicochemical properties of mutated amino acids on the resistance of penicillin binding proteins [8]. The mutation positions and various chemical descriptors were utilised as protein sequence and ligand descriptors, respectively.

The article "Proteochemometric Method for pIC50 Prediction of Flaviviridae" was published in 2022. Journal: Biomed Res Int.

### 1.2. Approach

In this work, we developed a PCM-based model for the prediction of pIC50 values for peptides against the Flaviviridae family. The peptides and target proteins were cumulatively studied using PCM descriptors which included peptide properties, z-scales for peptides, proteins, and peptide-protein interaction. The complete workflow of the study is shown in Figure 1.

The overall approach of the study includes:

- Curation of dataset
- Defining PCM descriptors
- Methodology and training of the machine learning model
- pIC50 prediction algorithm results

## 2. Materials and Methods

This section elaborates on data, features, and details of the machine learning algorithms.

### 2.1. Curation of the Dataset

The datasets are made up of publically available antiviral peptide data with their IC50 values and the target proteins collected from the literature. This results in two datasets:

- Antiviral peptides with IC50 values (Dataset 1) and
- Antiviral peptides with IC50 values and their target proteins (Dataset 2).

#### 2.1.1. Dataset 1

Antiviral peptide data is taken from the publicly available AVP-IC50 dataset [9]. The dataset consists of AVP sequences, IC50 values in micromolar and their respective viral families. From these, peptides for only the Flaviviridae family are taken, constituting Dataset 1 with total of 130 sequences.

#### 2.1.2. Dataset 2

For Dataset 2, along with the AVP, Flaviviridae target proteins are also taken. The target proteins of the antiviral peptides have been identified in the literature [10–30]. Here, 50 peptide sequences out of 130 have defined targets. These 50 peptide sequences along with their target protein sequences form Dataset 2. Target protein sequences are extracted from Uniprot [31].

#### 2.1.3. pIC50

The IC50 values in the datasets ranged from 0.001 micromolar to 440 micromolar making the distribution very skewed, as shown in Figure 2(a). This would have made it difficult for the model to extract informative patterns to learn from. Thus, the IC50 values were negative log transformed to give the pIC50 value. This is done using the following formula:

(1) $$\begin{array}{c} \text{pIC}50=-\ln\left(\text{IC}50*10^{-6}\right) \end{array}$$

The data distribution after converting to pIC50 is shown in Figure 2(b). Hereafter, pIC50 will be used in the rest of the paper.

The article "Proteochemometric Method for pIC50 Prediction of Flaviviridae" was published in 2022. Journal: Biomed Res Int.

### 2.2. Defining PCM Descriptors

PCM modeling works based on descriptors which are mathematical representations of various properties of peptides and their target proteins. Here, we are looking at the following descriptors which are calculated for peptides and their target proteins:

- Physicochemical properties of peptides and target protein
- Z-scale for peptides, target protein, and their cross-term

*Physicochemical properties*. Peptide and target protein properties were calculated from their amino acid sequences using Biopython package [32]

*Z-scales*. The peptides and target proteins used in this work are represented using five z-scale descriptors (*z*_1_, *z*_2_, *z*_3_, *z*_4_, and *z*_5_) of their amino acid as derived by Sandberg et al. [33]. The z-scale represents their hydrophobicity (*z*_1_), steric bulk properties and polarizability (*z*_2_), polarity (*z*_3_), and electronic effects (*z*_4_ and *z*_5_). These five z-scales are the principal components of 26 computed and measured physicochemical properties of amino acids. To get a z-scale descriptor for a peptide and protein, the average is taken of their amino acid z-scale vectors. The z-scale descriptors for both peptides and proteins are normalized to standard normal. In order to incorporate the information about the interaction between protein and the peptide, cross-term descriptors were also included. This is calculated as flattened out outer product of normalized peptide z-scales and normalized protein z-scales resulting in 25 (5x5) dimensional vector. As a result, each peptide-protein pair is represented as a 35 dimensional vector (5 peptide z-scale, 5 protein z-scale and 25 cross-term)

*Descriptor groups*. In order to perform various machine learning experiments, multiple groups of descriptors were created as defined as follows:

- Physicochemical properties for peptides (PP)
- Physicochemical properties for target protein (TP)
- Peptide z-scale descriptors (PZ)-5 z-scale descriptors calculated for peptide sequences
- Target protein z-scale descriptors (TZ)-5 z-scale descriptors calculated for target protein sequences
- Cross term descriptors (XZ)-Multiplication of peptide and target protein z-scale descriptors generated the cross term descriptors group

### 2.3. Machine Learning Details

In this section, we discuss the features selection method, machine learning algorithm, and evaluation criteria of the model.

*Feature selection*. In machine learning, it is important to have useful input features or descriptors. Therefore, in order to remove uninformative predictors, feature selection is carried out. This not only removes noise from the data, but also reduces dimensionality of the data which makes the trained model less complex and more interpretable. The feature selection for this work is carried out in two steps. First, the feature ranking is obtained using Recursive Feature Elimination. This is followed by adding the features iteratively starting from the highest ranking feature and checking for their predictive performance. Further, only those features were added to the final feature set whose addition improved the adjusted-*R*^2^ value. The calculation of adjusted-*R*^2^ based on *R*^2^ value is as follows:

(2) $$\begin{array}{c} \text{adjusted}-R^{2}=1-\frac{\left(1-R^{2}\right)\left(n-1\right)}{n-p-1}, \end{array}$$

where *R*^2^ is sample R-squared value, *n* is number of examples, and *p* is number of predictors.

The article "Proteochemometric Method for pIC50 Prediction of Flaviviridae" was published in 2022. Journal: Biomed Res Int.

*Random Forest*. Random Forest is an ensemble learning method for classification and regression. The underlying principle is to construct multiple decision trees and aggregate the output from each decision tree. In case of a regression problem, most common means of aggregating the output is mean of the predictions. In Random Forest, each of the decision tree is trained on a randomly selected subset of features and examples from the training data which causes each tree to learn different patterns from the same training data. This results in a reduced variance, making the model more effective. Random Forest regressor model from scikit-learn library [34] was used

*Evaluation criteria*. The selection of informative performance metrics is vital in order to measure effectiveness of a prediction model. Therefore, to informatively measure performance of the prediction models, performance measures used in this work is described as follows:

- Root Mean Squared Error (RMSE):

(3) $$\begin{array}{c} \text{RMSE}=\sqrt{\frac{1}{n}\underset{i}{\sum }{\left(y_{i}-{\overset{\wedge }{y}}_{i}\right)}^{2}} \end{array}$$

(ii) Mean Absolute Percentage Error (MAPE):

(4) $$\begin{array}{c} \text{MAPE}=\frac{1}{n}\underset{i}{\sum }\frac{\left|y_{i}-{\hat{y}}_{i}\right|*100}{y_{i}} \end{array}$$

(iii) R-squared value (*R*^2^):

(5) $$\begin{array}{c} R^{2}=1-\frac{SS_{res}}{SS_{tot}},\\ SS_{res}=\underset{i}{\sum }{\left(y_{i}-{\overset{\wedge }{y}}_{i}\right)}^{2},\\ SS_{res}=\underset{i}{\sum }{\left(y_{i}-\overset{¯}{y}\right)}^{2}, \end{array}$$

where *SS*_*res*_ is residual sum of squares, *SS*_*tot*_ is total sum of squares

(iv) Pearson's Correlation Coefficient (PCC):

(6) $$\begin{array}{c} PCC=\frac{\sum_{i}\left(y_{i}-\overset{¯}{y}\right)\left(\left({\hat{y}}_{i}-\overset{¯}{\hat{y}}\right)\right)}{\sqrt{\left(\sum_{i}{\left(y_{i}-\overset{¯}{y}\right)}^{2}\right)\left(\sum_{i}{\left({\overset{\wedge }{y}}_{i}-\overset{¯}{\hat{y}}\right)}^{2}\right)}}, \end{array}$$

where y is actual pIC50 value, $\hat{y}$ is predicted pIC50 value, $\overset{¯}{y}$ is mean of actual pIC50 values, and $\overset{¯}{\hat{y}}$ is mean of predicted pIC50 values

The article "Proteochemometric Method for pIC50 Prediction of Flaviviridae" was published in 2022. Journal: Biomed Res Int.

### 2.4. Methodology

This section elaborates on utilizing the curated data, properties, and algorithm for training the suitable model. As explained in 2.1, properties were calculated for Dataset 1 and Dataset 2. Dataset 1 was studied using physicochemical properties. However, for Dataset 2 all descriptor groups (as explained in Section 2.2) were calculated as they contain both peptide and target protein information. Using only the peptide properties for Dataset 1 to train the model, resulted in lower *R*^2^ value. Considering this, this study further focuses on utilizing Dataset 2.

We see an improvement in the results with the addition of peptide and target property groups in the model. Using multiple sequence descriptors can be helpful for the model to learn. Hence, along with properties, z-scales are used to represent the sequences. The model was trained on peptide (PZ) and target protein z-scales (TZ), which further improved the performance of the model. The PCM approach includes one more cross-term group (XZ). A combination of property groups for peptides (PP), target proteins (TP), and z-scale groups (PZ, TZ, and XZ) performs the best out of all the combinations. The descriptors calculated and the combinations are illustrated in Figure 1. Furthermore, in order to remove the noisy or noninformative features, we performed feature selection as explained in Subsection 2.3. During the feature selection phase, Random Forest with default parameters is used as a base regression model.

The Random Forest model is then tuned on the selected features to achieve the best performance. For this, we use the grid search approach where hyperparameters form the axis of the grid and each point on the grid is a combination of defined values for each hyperparameter. 5 fold cross-validation on Mean Absolute Percentage Error (MAPE) helps to obtain best performing hyperparameter values. The hyperparameters and their values for which the Random Forest model is tuned are mentioned in Table 1. As a last step, the Random Forest training is done on the best preforming feature set and hyperparameters, and its predictive performance is evaluated. Furthermore, to ensure fairness of the results, all performance measures are calculated using Leave-one-out (LOO) cross-validation (CV).

The article "Proteochemometric Method for pIC50 Prediction of Flaviviridae" was published in 2022. Journal: Biomed Res Int.

## 3. Results and Discussion

In this section we look at the results obtained for various combinations of descriptor groups. Results for some of the example sequences are mentioned in Table 2. It can be seen from the results that the predicted pIC50 values are very close to actual pIC50 values. The performance of the model is evaluated using Leave-one-out cross-validation and the results are tabulated in Table 3.

The model is trained using only peptide properties which resulted in the low R-squared value of 0.29 and high mean absolute percentage error of 17.10%. To understand this, we have done further analysis of the dataset. We observed that there are certain peptide sequences in the dataset which are very similar but still have very different pIC50 value and vice versa. Similar is the observation for physico-chemical properties based descriptors. This might make it difficult for the model to learn informative patterns from the peptides alone and needs additional information.

Based on the results in Table 3, the rest of the experimentation are performed using PCM approach. The addition of target protein properties improved the results in R-squared value of 0.30 and MAPE of 18.82. The combination of z-scale for peptide and protein significantly improved the results giving R-squared value of 0.72 and MAPE of 11.32%. The details of peptide and target protein combinations for z-scale and physicochemical properties are detailed in Section 2.2.

In PCM, along with the target and peptide descriptor groups, cross-term z-scales are often considered as they represent the potential of peptide and target protein. The model has been trained using the three descriptor groups (PZ, TZ, and XZ). The addition of peptide protein cross-term descriptor slightly improved the predictive performance of the model further, giving R-squared value of 0.76 and MAPE of 9.48%.

The best results with R-squared value of 0.85 and MAPE of 8.44% are obtained with combinations of z-scale and physicochemical properties.

### 3.1. Discussion

Despite various scientific discoveries and advancements, viruses continue to be one of the threats to human health [35]. Antiviral peptides (AVPs) are emerging as one of the interesting alternative therapeutics to viral concerns. Although elusive, antiviral peptides do exhibit certain physicochemical properties which makes them great candidates for antiviral therapeutics [1]. The work done by Surana et al. explains the usage of physicochemical properties [36]. Although physicochemical properties do help in identifying the potential antiviral peptides, IC50 is one of the methods used for further validating the efficacy of candidate peptides [37]. In order to predict the candidate peptides as close to the experimental method as possible, we propose the prediction of pIC50 in our current study.

The article "Proteochemometric Method for pIC50 Prediction of Flaviviridae" was published in 2022. Journal: Biomed Res Int.

We initially utilized a combination of peptide properties and IC50 of known peptides to create the algorithm. However, we discovered that there is no direct correlation between the peptides and the IC50 values. The behavior of a peptide depends on its own properties as well as the nature of the target against which the peptide is going to act. This is where PCM methods seem to be the right approach because it does not only take the peptides but also takes the target protein into account.

PCM models give the flexibility to study multiple ligands (peptide in this case) and multiple target setups, which become beneficial in the current study. As for Flaviviridae AVPs, although they are all against flaviviruses, they have different targets that they act upon. As explained earlier, the major features utilized were the physicochemical properties of peptides and target proteins. We observed that adding the physicochemical properties of target proteins improved the pIC50 prediction for the peptides. Along with the basic physicochemical properties, the addition of Z-scores gave a boost to the model performance.

The Z-score includes the hydrophobicity, steric bulk properties, polarity, polarizability, and electronic effects giving additional features to the physicochemical properties. The Z-scores individually cover the features of peptides, target proteins, and cross-descriptors covering the interaction features between the peptide and target proteins. The cross-terms features give an additional edge in terms of covering the ligand-target interactions instead of only features of individual peptides and targets. Multiple combinations of physicochemical properties and Z-score descriptors lead us to the model with the best descriptors giving good predictions. The best descriptors identified were target polarity, cross-term of peptide polarity, and target hydrophobicity along with aromaticity. It can be inferred that aromaticity, along with hydrophobicity and polarity of protein and peptide, best describes the relationship and hence the prediction of IC50.

We further explored the PCM2Vec methodology for IC50 predictions. However, we did not get very good results there, and it needs to be explored further. PCM2Vec can be a promising algorithm which can be explored in future work.

## 4. Conclusion

In this study we have applied proteochemometric modeling to study the pIC50 values for AVPs against the Flaviviridae family. The activity prediction of probable antiviral peptide brings in additional validation to the efficacy of AVP to choose the peptide for further experiments based on their pIC50 value, and thus reducing the time and cost for the experimental cycle. As most of the peptides or drug candidates are built against specific targets, being able to predict their bioactivity values is one step closer to getting more accurate peptides. This can be further extended to multiple viral families or target-based PCM models. Currently we have considered entire target sequences, however, further study can be done to include binding site residues and their interactions. Taking binding site residues into consideration might further boost the algorithm performance.

The article "Proteochemometric Method for pIC50 Prediction of Flaviviridae" was published in 2022. Journal: Biomed Res Int.

## Figures and Tables

**Figure 1:** PCM model flowchart. Illustration of the descriptors and multiple combinations of descriptor groups used to predict the pIC50 using Random Forest.

**Figure 2:** Distribution of IC50 and pIC50 values.

**Table 1:** Range of values used to tune hyperparameters for Random Forest.

Hyperparameter	Ranges
n_estimators	100, 200, 250, 300, 500, 1000, 1500
min_samples_split	2, 5, 10
min_samples_leaf	1, 2, 4
max_features	auto, sqrt, log2
max_depth	2, 3, 5, 10, 15, 20, None
bootstrap	True, False

**Table 2:** Actual and predicted pIC50 values for example sequences.

Sequence	Actual pIC50 value	Predicted pIC50 value
AFLGWIGAIVSTALPQWR	11.289	11.261
ACFPWGNTWCGGK	11.250	11.262
MANAGLQLLGFILAFLGWIGAI	12.429	11.224
RWMVWRHWFHRLRLPYNPGK NKQNQQWP	11.736	11.246
AAQRRGRIGRNPSQVGD	7.934	8.158
RTGRGRRGIYR	10.271	11.294
GELGRLVYLLDGPGYDPIHCSL AYGDASTLVVF	17.678	19.780

**Table 3:** Results of obtained models.

Descriptor combinations	*R* ^2^	MAPE	PCC	MSE
PP	0.48	14.04	0.72	6.88
PP+TP	0.72	11.46	0.84	3.70
PZ+TZ	0.72	11.32	0.85	3.63
PZ+TZ+XZ	0.76	9.48	0.87	3.14
PP+TP and PZ+TZ+XZ	**0.85**	**8.44**	**0.92**	**1.99**

## Data Availability

The code and data is available at https://github.com/thoughtworks/mic-predictor
